# Observation and Analysis of the Postoperative Analgesic Effect of Subanaesthetic Dose of Ketamine in Kashin–Beck Disease Patients after Total Knee Arthroplasty

**DOI:** 10.1155/2022/9417594

**Published:** 2022-02-25

**Authors:** Huijin Xie, Gaobo Zhu, Changmou Zhu, Wei Wang

**Affiliations:** ^1^1 Emergency and Trauma Surgery, The First College of Clinical Medical Science, China Three Gorges University, Yichang 443003, China; ^2^2 Emergency and Trauma Surgery, Yichang Central People's Hospital, Yichang 443003, China

## Abstract

With the transformation of modern medical models, the medical needs of patients have changed from treatment to safe, comfortable, and painless treatment. Therefore, it is clinically important to find an ideal analgesia model to reduce the pain after total knee arthroplasty and minimize the impact of surgical trauma on the body pressure. This article aims to study the effects of lower limb nerve block combined with local infiltration analgesia of the joint cavity on the hemodynamics and postoperative analgesia effects of knee joint replacement in elderly patients by comparing the effects of the subanaesthetic dose of ketamine on the hemodynamics and postoperative analgesia effect of knee joint replacement in elderly patients' intraoperative analgesia program. This article proposes that 90 patients requiring unilateral total knee replacement were randomly divided into 3 groups, with 30 patients in each group, age 65–85 years, average age 75 years, ASA I ∼ II grade, and body mass index 13.89 ∼ 37.26. Use a multifunctional monitor to monitor the patient's continuous blood pressure (SBP/DBP) and mean arterial pressure (MAP), heart rate (HR), electrocardiogram (ECG), intraoperative pulse oxygen saturation (SpO_2_), and end-tidal carbon dioxide (PETCO_2_). The following are monitored: record the heart rate (HR), systolic blood pressure (SBP), and diastolic blood pressure before induction of anesthesia (T0), before the upper tourniquet (T1), and after the upper tourniquet (T2), before tourniquet withdrawal (T3), and after tourniquet withdrawal (T4), mean arterial pressure (MAP). The three groups of patients had different degrees of itching, vomiting, nausea, and other adverse reactions. The experimental results in this article show that, in elderly patients with epidural anesthesia, the use of propofol and dexmedetomidine to maintain the patient's BIS value between 60 and 70 can meet the depth of sedation required for surgery without important surgical operation knowledge.

## 1. Introduction

With the ever-changing medical standards and the continuous improvement of people's living standards, people's requirements for the quality of life and perioperative comfort have also been further improved. The concept of rapid recovery surgery that minimizes perioperative pain and trauma is becoming the future development direction of medical treatment and has also put forward greater requirements and challenges for anesthesiologists. A common early complication after surgery or anesthesia is postoperative cognitive dysfunction (POCD). Cognitive disorders such as stress, personality changes, memory loss, and inability to concentrate after surgery or anesthesia can lead to mental confusion and reduce social behavior ability in severe cases. On the premise of ensuring the safety of patients' lives, we will further protect the cognitive function of patients, reduce the brain damage caused by anesthesia and surgery, improve the comfort of patients during the perioperative period, and accelerate the recovery of patients after surgery. We need to make continuous attempts and work hard.

With the clinical development and advancement of joint replacement technology, total knee arthroplasty (TKA) technology has developed rapidly in recent years, has become an important treatment method for the treatment of end-stage KOA, and has gradually formed a medical industry. The consensus has also been recognized by many patients. Research and observation by many clinicians at home and abroad have shown that TKA can quickly and effectively eliminate patients' joint pain symptoms and improve or even fully restore joint function. However, joint replacement surgery is different from other orthopedic surgeries in that it requires early functional exercise after the knee. However, due to the large trauma, the patient's early postoperative pain symptoms are the most obvious, and even severe and unbearable pain will affect the patient's body and mind. It causes a series of negative effects and hinders the early functional exercise of the joints of patients, reducing the efficacy of surgery. Some scholars have also pointed out that severe pain may even be accompanied by respiratory complications and incision infections. Therefore, the pain after TKA has attracted the attention and concern of many clinicians. Relieving postoperative pain can not only reduce the patient's pain and improve the patient's satisfaction with the operation but also enhance the patient's confidence to exercise joint function early.

The key contributions of this work are as follows:

1. Previous studies of total knee arthroplasty analgesia focused on the feasibility of postoperative analgesia. This experiment started from specific clinical populations and selected elderly patients as the research objects, focusing on the surgical operation analgesia. The safety and effectiveness of postoperative analgesia programs provide a theoretical basis for the choice of anesthesia and analgesia methods for this group during the perioperative period.
2. The wireless communication energy consumption model is proposed, and the Raft consensus algorithm design based on clustering and the distance measurement in cluster analysis, the medical IoT, and data fusion technology are used to observe and analyze the neuroprotective total knee of patients with Kashin–Beck disease and provide technical support for the postoperative analgesic effect of the subanesthetic dose of ketamine in joint replacement surgery.

## 2. Related Work

Martin presented the benefits of injecting caquester into the joints of patients who were resolved after the seat frame was fixed. His study included 64 patients with rheumatoid arthritis who also underwent initial total knee arthroplasty [1]. The term “large knee surgery” includes anterior cruciate ligament reconstruction, knee lysis, and total knee replacement. Freytes study found that although the current surgical techniques have been improved, postoperative pain in these operations is still a problem. There are several analgesic options, each with its own characteristics, but still, there is a lack of consensus on the best method for postoperative pain in this type of surgery. Provide available evidence on current major knee surgery analgesia techniques, with emphasis on total knee replacement and regional anesthesia. In order to better understand different nerve block techniques, a brief anatomical review is also given. Searches were made in medical databases (PubMed and Cochrane) and anesthesiology journals (including *Regional Anesthesia and Pain Medicine*, *Journal of Anesthesiology*, and *British Journal of Anesthesiology*) [2]. Although there is little evidence of risks and benefits, it is increasingly advocated for patients to self-medicate during hospitalization. It is well known that pain control after total knee arthroplasty (TKR) is poor. The purpose of Deane's study is to determine whether patients undergoing TKR surgery who self-administer oral analgesics immediately after surgery have better pain control (treatment as usual) than patients who receive pain control through a nurse-led medication round (TAU). A prospective, parallel design, open-label, and randomized controlled trial compared patient-guided pain self-management after TKR and nurse-controlled oral analgesia (TAU) for pain control [3]. Although the research perspective is forward-looking, there are still many unachievable parts of the technology.

## 3. Medical IoT and Its Data Fusion Technology

The medical IoT is the application of advanced IoT technology to medical enterprises. As my country's medical and health system evolves from clinical information to regional, medical, and health information, the IoT technology has matured: to solve people's concerns about their own health, the situation requires further promotion of medical care, and the development of the health information industry [4–7]. The network process of the medical IoT is shown in Figure 1.

### 3.1. Wireless Communication Energy Consumption Model

At this time, there are more obstacles, and they cause greater interference, and the energy consumption will increase sharply as the distance increases [8–10]. It can be seen that when the distance between nodes is *d*, the energy consumption *E*_*r*_ required to transmit *K* bits of information is as follows:

(1) $$\begin{array}{c} E_{r}=\left\{\begin{array}{cc} kE_{\text{elec}}+k\varepsilon d^{2}, & d<d_{0},\\ kE_{\text{elec}}+k\varepsilon_{\text{mp}}d^{4}, & d\geq d_{0}, \end{array}\right. \end{array}$$

in which *E*_elec_ represents the energy consumed by the wireless transceiver circuit, which mainly depends on digital coding and filters [11, 12]; *εd*^2^ and *ε*_mp_*d*^4^ represent the energy consumed by the signal amplifier to transmit each bit of data; *k* represents the data length of the packet [13, 14]; *d* represents the distance between nodes; *d*_0_ represents the threshold of energy consumption for communication. *E*_*r*_ is the energy consumption of the received signal, and the formula is

(2) $$\begin{array}{c} E_{r}=kE_{\text{elec}},\\ E_{r}=k\left(E_{\text{elec}}+E_{\text{df}}\right). \end{array}$$

The standard hard threshold at initialization is expressed as

(3) $$\begin{array}{c} {\text{NHT}}_{\text{initial}}=\text{HT}-\text{ST}. \end{array}$$

When initializing, the nodes in the network are in a dormant state [12, 15]. Only when the monitoring data meet condition (4) can the node be active, enter the state of receiving and sending data, and update the NHT value to the monitored data value [16]. Among them, the monitoring data are represented by MD.

(4) $$\begin{array}{c} \text{MD}>\text{HT}\&\&\left|\text{MD}-\text{NHT}\right|\geq \text{ST}. \end{array}$$

For nodes that have been activated, they can send and receive data. When condition (5) is met, the value of NHT is updated to MD, and then its data value is transmitted to the upper node.

(5) $$\begin{array}{c} \text{MD}>\text{HT}\&\&\left|\text{MD}-\text{NHT}\geq \text{ST}\right|. \end{array}$$

### 3.2. Raft Consensus Algorithm Based on Clustering

Among them, *n* represents the bandwidth, *K*(*x*) represents the kernel function, and *k*(*x*) satisfies the following conditions:

(6) $$\begin{array}{c} f_{n}\left(x\right)=\frac{1}{h}\sum_{i=1}^{h}K_{n}\left(x-x_{i}\right)=\frac{1}{nh}\sum_{i=1}^{h}K\left(\frac{x-x_{i}}{n}\right),\\ K\left(x\right)\geq 0,\\ \int K\left(x\right)\text{d}x=1,\\ \int^{}xK\left(x\right)=0,\\ \int x^{2}K\left(x\right)\text{d}x>0,\\ \text{MISE}\left(h\right)=E\int {\left(f_{n}\left(x\right)-f\left(x\right)\right)}^{2}\text{d}x,\\ \text{AMISE}\left(n\right)=\frac{R\left(K\right)}{nh}+\frac{1}{4}m_{2}K^{2}n^{4}R\left(f\right), \end{array}$$

in which

(7) $$\begin{array}{c} R\left(g\right)\int g{\left(g\right)}^{2}\text{d}x,\\ m_{2}\left(K\right)=\int x^{2}K\left(x\right)\text{d}x. \end{array}$$

In order to minimize MISE(*h*), it is transformed into a pole finding problem:

(8) $$\begin{array}{c} \frac{\partial }{\partial h}\text{AMISE}\left(n\right)=\frac{R\left(K\right)}{nh}+m_{2}K^{2}n^{3}R\left(f\right)=0. \end{array}$$

However, kernel density estimation cannot determine the optimal parameter in the example, but can reasonably determine the value range of the parameter [17].

### 3.3. Distance Measurement in Cluster Analysis

Many clustering algorithms divide data objects into different clusters by similarity. The similarity between clusters is low, and there is a high degree of similarity between cluster objects [18, 19]. The target distance is usually used as an index to measure the degree of target dissimilarity. Common distances are as follows:

(1) Euclidean distance:
  (9) $$\begin{array}{c} d\left(x_{i},x_{j}\right)=\left\|x_{i}-x_{j}\right\|={\left[\sum_{k=1}^{m}{\left|x_{ik}-x_{jk}\right|}^{2}\right]}^{1/2}. \end{array}$$
(2) Manhattan distance:
  (10) $$\begin{array}{c} d\left(x_{i},x_{j}\right)=\sum_{k=1}^{m}\left|x_{ik}-x_{jk}\right|. \end{array}$$
(3) Chebyshev distance:
  (11) $$\begin{array}{c} d\left(x_{i},x_{j}\right)=\text{max}\left|\underset{1\leq k\leq m}{x_{ik}}-x_{jk}\right|. \end{array}$$
(4) Minkowski distance:

(12) $$\begin{array}{c} d\left(x_{i},x_{j}\right)={\left[\sum_{k=1}^{m}{\left|x_{ik}-x_{jk}\right|}^{n}\right]}^{1/n}, \end{array}$$

in which *n* ∈ [l, ∞); when *n* = 1, it is the Manhattan distance, when *n* = 2, it is the Euclidean distance, and when *n* ⟶ ∞, it is the Chebyshev distance.

## 4. Analgesia after Total Knee Arthroplasty

### 4.1. Materials and Methods

#### 4.1.1. General Information

The techniques involved in this research are all routine techniques in the scope of clinical anesthesia in our hospital, which do not increase the hospitalization costs of patients and have less traumatic stimulation and operation for patients [20, 21]. The personal information collected in the experiment is only used in this clinical study and is used before the experiment. The experimenter informs the test patients and their families of the research purpose, plan, and possible risks, and all the test patients have signed an informed consent form [22, 23]. A total of 90 patients were included in this study. There were no significant differences in general data such as gender, age, height, weight, BMI value, and ASA classification among the three groups of patients. The comparison of the general conditions of the three groups of patients is shown in Table 1.

#### 4.1.2. Inclusion and Exclusion Criteria

The inclusion criteria were as follows: patients undergoing elective bilateral total knee replacement surgery in an affiliated hospital from June 2019 to May 2020, regardless of gender, age 60–75, ASA classification I-II, and BMI no more than 30 kg/m^2^.

### 4.2. Research Methods

All subjects were abstained from eating and drinking for 8 hours before the operation. In order to avoid the error of the research results caused by other drugs, all the patients did not use the preoperative medication. After entering the room, the patient was given routine monitoring (ECG, heart rate, and oxygen saturation), peripheral venous catheterization, established unobstructed venous access, and intravenous infusion of sodium lactate solution 10–15 ml/kg. The patient was given oxygen inhalation with a mask, and the oxygen flow rate was 3 L/min. In order to monitor the patient's blood pressure more accurately and closely, a radial artery perforation catheter connected to a disposable pressure sensor is provided for the patient to monitor invasive blood pressure (ABP). After cleaning the patient's forehead and face with 75% alcohol, connect the front electrode of the dual-frequency EEG monitor, and use the dual-frequency EEG indicator (BIS) to detect the patient's depth of inhibition. This operation requires the use of bone cement to shape. During the operation, the room temperature must be kept low. The surgical wound is large. The patient is often accompanied by severe body temperature loss. We adopt intraoperative temperature monitoring and use a body surface temperature probe to continuously monitor the patient's axillary temperature. If the patient's axillary temperature is below 36.0°C, we will use a fan heater to keep warm, and 38.0°C warm air will be blown through the shoulder to raise the patient's body temperature.

Epidural anesthesia: all patients choose the L2-3 or L3-4 puncture point for epidural anesthesia, the tip is placed with a tube, the depth of which is 2–4 cm, the catheter is fixed, and no blood and cerebrospinal fluid are drawn back; the experimental amount is given as 2% lidocaine 3 ml, and 5 minutes later, observe whether the patient has the phenomenon of local anesthetic entering blood and general spinal anesthesia. The additional concentration is 2% lidocaine 6 ml and ropivacaine 4 ml. The block level will be tested after 5 minutes of additional medication. Adjust the amount of the epidural drug to control the patient's block level below T8. After the anesthesia is satisfied, start disinfection, spread a sterile excipient sheet, and add 5 ml of ropivacaine via an epidural tube every 1 h after the administration is over.

Sedation method: preexperimental results show that bilateral knee joint replacement requires approximately 15 minutes for disinfection and sterilization. In the dexmedetomidine group (group D), 5 ug/ml of dexmedetomidine was intravenously infused when the lower limbs were disinfected. The suction load was about 0.8 ug/kg within 15 minutes, and the pumping speed was adjusted to 0.2–0.8 ug kg^−1^ h^−1^. The propofol group (P group) started to be administered at the same time as the start of the competition. Propofol 1 mg/kg was injected intravenously within 1 minute, and then the propofol pump 1–4 mg kg^−1^ h^−1^ was continuously injected. The group adjusted the injection speed of the infusion pump according to the BIS value and checked that the BIS value was between 60 and 70. Both groups stopped pumping sedative drugs when the second knee joint capsule was sutured.

### 4.3. Observation Index and Index Evaluation Standard

After the operation, the three groups of patients were recorded by the same ward nurse in the same single-blind method to record the visual analogue scale (VAS) scores for 2 h, 4 h, 6 h, 12 h, and 24 h after surgery: painless, 10 for drama pain; <3 is excellent, 3-4 points and ≥5 points. At the same time, the patients were invited to make a comprehensive evaluation of the preemptive analgesia plan. There are 5 levels: level I, excellent; level II, very good; level III, good; level IV, fair; level V, poor. Sensory block recovery time is carried out at the same time: after the operation, acupuncture is used and measured every 10 minutes, and the skin sensory recovery time of the Tio-L1 spinal nerve innervation area is used as an indicator: the recovery time of motor block, measured once every 10 minutes. Respiratory depression refers to breathing <10 bpm or SPO_2_ <95%.

## 5. Experimental Results and Observation Analysis

The operation time of all tested patients was greater than 1 h and less than 3 h. There was 1 case in group D with intraoperative blood transfusion, and there were 2 cases in group P. No statistical difference was found in blood transfusion (*P* > 0.05).

### 5.1. Comparison of Intraoperative Vital Signs

First, we compared the average levels of MAP, HR, and SPO_2_ at four different time points of the two groups of patients at T0, T1, T2, and T3. From the overall level, we found that there was no significant difference in MAP and HR between the two groups of patients at T0. The MAP after external anesthesia and sedative pump injection was significantly lower than that at T0 (*P* < 0.01). Comparing the MAP levels of the two groups of patients at T1, T2, and T3, we found that the difference between group P and group D was significant (*P* < 0.01), and group P was smaller than group D. After pumping dexmedetomidine in group D, the heart rates of T1, T2, and T3 were significantly lower than those at T0 (*P* < 0.01), while the propofol group did not have such a performance; comparing the HR of the two groups of patients at T1, T2, and T3, it was found that the heart rate of patients in group D was significantly lower than that in group P (*P* < 0.01). After sedation, the SPO_2_ values of the two groups were lower than T0, but there was no significant difference between the two groups (*P* > 0.05).  Table 2 shows the comparison of MAP, HR, and SPO_2_ between the two groups of patients at different times.

#### 5.1.1. Blood Sugar

24 hours after the operation, blood glucose of the three groups reached the highest value, and blood glucose of the patients in the C and S groups basically returned to normal. The three time points of T1, T2, T3, and T4 in group F had significant differences between the three time points of T1, T1, T2, T3, T5, T1, T3, and T5 (*P* < 0.05). Preoperative and postoperative changes of blood glucose concentration in the three groups are shown in Figure 2.

#### 5.1.2. General Conditions during Surgery

Intraoperative general conditions: there was no significant difference in the operation time and upper tourniquet time between the three groups of patients (*p* > 0.05); the dosage of sufentanil in group C (41 ± 8.5 ug) was compared with group S (38.5 ± 8.5 ug). The comparison of the intraoperative conditions of the three groups of patients is shown in Table 3.

#### 5.1.3. Tumor Necrosis Factor-*α* (Normal Reference Value: 0.74–1.54 ng/ml)

The changes of TNF-*α* concentration in the three groups before and after surgery are shown in Figure 3.

#### 5.1.4. Comparison of Diastolic Blood Pressure

At T2, the difference in DBP between group F and group C was statistically significant (*p* < 0.05). The comparison of intraoperative DBP changes in the three groups of patients is shown in Table 4.

#### 5.1.5. Angiotensin II (Normal Reference Value: 28–115 pg/ml)

The concentration of angiotensin II and all three groups began to increase when the skin was cut and reached a peak after bone cement was placed. After 24 h, the Ang-II concentration of T1, T2, and T3 groups and the Ang-II concentration of the F group were significantly different in the T1, T2, and T2 groups compared with those before operation (*P* < 0.01). Compared with group F, group C and group S have extremely significant differences in T1, T2, T3, and T4 angiotensin II (*P* < 0.01); group B and group C are compared at T1, T2, T3, and T4. There are significant differences (*P* < 0.05).  Figure 4 shows the changes in the levels of angiotensin in the three groups of patients before and after surgery.

### 5.2. Comparison of Postoperative Analgesia in Patients

The VAS scores of group F were higher than those of groups C and S within 24 hours after operation, and the difference was significant (*P* < 0.05 or *P* < 0.01). The difference between group C and group S at 6 h and 12 h after surgery was very significant (*P* < 0.01). The patient's pain trend change at rest is shown in Figure 5.

By comparing the postoperative VAS scores and trend changes of patients in the resting state and in the exercise state, the results showed that the median postoperative VAS score in group F was 2 (1) at 8 h, 12 h, and 24 h after the operation in the exercise state. ,2), 3(2,3) and 4(2,4) and the median VAS scores of group S 2(2,2), 3(2,3) and 4(3,5) compared with group C VAS The median scores of 3(2,3), 4(4,5) and 5(3,6) were significantly reduced (*p* < 0.05).  Table 5 shows the comparison of the VAS scores of the three groups of patients in the postoperative exercise state.

### 5.3. Comparison of Postoperative Adverse Reactions

At T2, the MAP difference between group F and group C was statistically significant (*p* < 0.05), while group S and group C had no significant difference in MAP (*p* > 0.05). The comparison of intraoperative MAP changes in the three groups of patients is shown in Table 6.

There was no significant difference in the preoperative heart rate of the three groups of patients (*p* > 0.05). There was no significant difference in the heart rate before and after the tourniquet was removed (*p* > 0.05). After the tourniquet was applied, the HR difference between group F and group C was statistically significant (*p* < 0.05); after the tourniquet was applied, the HR of group S was not significantly different from that of group C, and it was not statistically significant (*p* > 0.05). The comparison of intraoperative HR changes in the three groups of patients is shown in Figure 6.

In groups F, S, and C, the incidences of postoperative nausea and vomiting were 13.4%, 10%, and 16.7%, and the incidences of irritability were 6.7%, 6.7%, and 10%, respectively. There was no statistically significant difference between the groups (*p* > 0.05). The postoperative adverse reactions of the three groups of patients are shown in Table 7.

## 6. Conclusions

The results of this study showed that preoperative ketamine combined with clonidine epidural block significantly prolonged the recovery time of sensory and motor nerve blocks. Clonidine is used in combination with local anesthetics for peripheral nerve block. Its analgesic site is in the epidural space of the spinal cord. The most common complications of epidural block are nausea and vomiting. Ketamine and bone cement also have this side effect. However, there was no difference in the incidence of PONT between the three groups in this study, which may be related to the regular use of ondansetron after surgery and the excellent analgesic and sedative effects of preventive analgesia. In addition, the incidence of side effects of ketamine is related to the dose and mode of administration, and the incidence of intravenous and intramuscular administration is higher. In this study, low-dose epidural ketamine may not cause obvious side effects of nausea and vomiting. The main side effect of ketamine is psychiatric symptoms, which mainly occur when used alone or when the dose is too high. A large number of studies at home and abroad have confirmed that plasma ketamine levels below 50 ng/ml will not cause hallucinations or cognitive impairment. The main side effects of clonidine are hypotension, sedation, and lethargy. Anesthetic dose of ketamine (intravenous dose <0.5 mg/kg, mainly 0.1–0.5 mg/kg) has an analgesic effect, has a short duration, and has almost no related side effects. It is suitable for short-term outpatient surgery and has no obvious effect on the patient's breathing. The inhibitory effect of this type of anesthesia ensures more stable hemodynamics and the safety of this type of anesthesia to maintain spontaneous breathing.

## Figures and Tables

**Figure 1:** Network process of the medical IoT.

**Figure 2:** Changes in blood glucose concentration of the three groups of patients before and after surgery.

**Figure 3:** The changes of TNF-*α* concentration in the three groups of patients before and after surgery.

**Figure 4:** Changes of angiotensin concentration in the three groups of patients before and after surgery.

**Figure 5:** Changes in the patient's pain trend at rest.

**Figure 6:** Comparison of intraoperative HR changes in the three groups of patients.

**Table 1:** Comparison of the general conditions of the three groups of patients $\left(\bar{X}\pm s\right)$.

Group	F group	S group	C group
Number of cases	30	30	30
Male/female	11/19	12/18	16/14
Age (years)	73 ± 5	75 ± 6	76 ± 5
Height (cm)	161.7 ± 10.3	167.10 ± 10.4	164.40 ± 9.8
Weight (kg)	58.6 ± 12.7	68.7 ± 15.3	65.2 ± 15.3
BMI (kg/m^2^)	22.5 ± 4.5	24.6 ± 5.0	25.2 ± 5.6
ASA classification (example, II/III)	11/19	14/16	9/21

**Table 2:** Comparison of MAP, HR, and SPO_2_ between the two groups of patients at different times $\left(\bar{X}\pm s\right)$.

Index	Grouping	T0	T1	T2	T3
MAP	Group F	106.88 ± 12.25	99.20 ± 12.30	98.60 ± 10.62	97.08 ± 10.31
	Group C	109.12 ± 12.30	95.92 ± 11.67	91.96 ± 11.21	91.88 ± 9.07
HR	Group F	77.20 ± 5.77	72.72 ± 5.34	67.60 ± 5.36	70.34 ± 7.03
	Group C	76.92 ± 5.55	74.40 ± 6.05	71.84 ± 5.54	74.48 ± 5.73
SPO_2_	Group F	100.00 ± 0.00	99.56 ± 0.51	98.48 ± 1.04	98.50 ± 1.06
	Group C	100.00 ± 0.00	99.36 ± 1.36	98.14 ± 1.08	98.10 ± 1.32

**Table 3:** Comparison of intraoperative conditions of the three groups of patients $\left(\bar{X}\pm s\right)$.

Group	F group	S group	C group
Operation time (min)	117.60 ± 17.70	120.70 ± 17.30	114.40 ± 16.80
Tourniquet time (min)	71.40 ± 9.70	73.50 ± 1130	76.50 ± 12.30
Sufentanil dosage (ug)	37.50 ± 9.502	38.50 ± 8.50	41.00 ± 8.50

**Table 4:** Comparison of intraoperative DBP changes in the three groups of patients.

Group	F group	S group	C group
T0	93 ± 15	92 ± 13	92 ± 13
T1	58 ± 10	60 ± 8	60 ± 8
T2	77 ± 11	88 ± 8	84 ± 10
T3	75 ± 11	74 ± 8	74 ± 10
T4	73 ± 12	70 ± 9	71 ± 11

**Table 5:** Comparison of VAS scores in the three groups of patients under postoperative exercise.

Group (h)	F group	S group	C group
2	2 (1, 2)	2 (1, 2)	2 (1, 2)
8	2 (1, 2)	2 (2, 2)	3 (2, 3)
12	3 (2, 3)	3 (2, 3)	4 (4, 5)
24	4 (3, 4)	4 (3, 5)	5 (3, 6)

**Table 6:** Comparison of intraoperative MAP changes in the three groups of patients.

Group	F group	S group	C group
T0	109 ± 16	110 ± 15	109 ± 13
T1	73 ± 10	74 ± 7	75 ± 8
T2	94 ± 11	105 ± 8	106 ± 9
T3	91 ± 11	90 ± 7	90 ± 12
T4	84 ± 12	83 ± 9	83 ± 13

**Table 7:** Postoperative adverse reactions in the three groups.

Group	F group	S group	C group
Nausea	2(6.7)	2(6.7)	3(10)
Vomiting	2(6.7)	1(3.3)	2(6.7)
Irritability	2(6.7)	2(6.7)	3(10)

## Data Availability

The data used to support the findings of this study are available from the corresponding author upon request.
